# A New Method for Early Screening of Gastric Cancer (G17 and CA724 Dual-Labeled Time-Resolved Fluorescence Immunoassay)

This article has been retracted.

**DOI:** 10.1155/2022/1704948

**Published:** 2022-07-20

**Authors:** Chang Liu, Cuicui Chen, Hongrui Lai, Huankun Liang, Shuhai Zhong, Guiling Guo, Lei Wang, Laiqing Li

**Affiliations:** ^1^Heilongjiang Academy of Chinese Medicine Sciences, Harbin, 150036, China; ^2^Guangzhou Youdi Bio-Technology Co., Ltd., Guangzhou 510663, China

## Abstract

Gastric carcinoma (GC) is one of the most common malignancies in the world with the great early screening challenges. The study is aimed at establishing a new detection method for early screening GC using time-resolved fluorescence immunoassay (TRFIA) via quantitative detection of gastrin-17 (G-17) and carbohydrate antigen 724 (CA724) in serum. Time-resolved analyzer measured the fluorescence intensity. The standards of G-17/CA724 were used for drawing the standard curve, which is used to calculate the concentration of G-17 and CA724 in serum sample. The sensitivity for G-17 was 0.54 pg/mL and for CA724 was 0.28 U/mL with a wide-range analyze concentration (0.1-1000) pg/mL or U/mL. The average recoveries ranged from 100.52% to 110.30% for G-17 and 103.02% to 116.00% for CA724. All CVs of the intra- and interassay were below 10% with high specificity. There was a high *Pearson* coefficient between this TRFIA method and the commercially available kits (Pearson *r* 0.9117 for G-17 and 0.9449 for CA724). Additionally, the cutoff value was 88.41 pg/mL and 5.47 U/mL for CA724 in health subjects. This study established a TRFIA method for simultaneous detection of the concentrations of G-17 and CA724 in serum, which provide a new method for sensitive, accurate, and specific early screening of gastric cancer.

## 1. Introduction

Gastrin is a circulating hormone produced by G cells in the gastric antrum. In addition to being responsible for initiating the release of gastric acid in response to food and/or body fluid factors, it also plays a role in the growth and maintenance of gastric epithelium, gastric mucosa, enterochromaffin-like cells, and gastric cancer [1, 2]. Gastrin and its precursors promote proliferation in different gastrointestinal cells. Hypergastrinemia resulting from atrophic gastritis and pernicious anemia leads to tumor formation in humans [3]. Mature, amidated gastrin-17 (G-17) can induce protein, mRNA expression, and transcription of the G1-specific marker cyclin D1, in the gastric adenocarcinoma cell line AGSE [4]. In particular, G-17 can be used as the “serological gastric biopsy” detecting multifocal atrophic gastritis [5]. Recent research has also demonstrated that G-17 is closely associated with GC progress, and it can promote GC cells invasion, proliferation, and migration in a dose-dependent fashion [6].

Carbohydrate antigen 724 (CA724) is the most sensitive and specific indicator for gastric cancer (GC) [7, 8]. Higher serum concentrations of CA724 are positively related to TNM stage, distant metastasis, recurrence, and poor overall survival [9, 10]. A meta-analysis suggested that the test of serum CA724 could do the best sensitivity and acceptable for the detection of GC particular among Chinese [11].

Biomarkers are biological molecules that are involved entirely or partially in carcinogenesis processes and, accordingly, can highlight abnormal changes in the patient [12] . Ideally, they should be noninvasive, sensitive, specific, cost-effective, and easy to implement in clinical routine. Taking this into account, liquid biopsy represents a good approach to achieve this objective. In this context, blood, urine, stool, saliva, or gastric juice could be interesting fluids to find new noninvasive biomarkers. In this review, a brief updated overview of potential noninvasive biomarkers for GC screening and early diagnosis is discussed [13] .

Early/primary screening of the patients with atrophic gastritis and early gastric cancer by endoscopy is unrealistic, and noninvasive serological screening is a practical method and should be further validated [14]. Time-resolved fluorescence immunoassay (TRFIA) is a novel detection technique with high sensitivity, lower matrix interference, and enlarge dynamic range, and it has been used in the diagnosis and screening of various human diseases [15–17]. However, TRFIA has not yet been used in G-17 and CA724 detection. Based on the roles of G-17 and CA724 on predicting atrophic gastritis and GC, we optimized and established a TRFIA method to detect the concentrations of G-17 and CA724, and it has the equivalent screening performance compared with clinical kits, which provide a new method for sensitive, accurate, and specific early screening of gastric cancer.

## 2. Materials and Method

### 2.1. Antigen, Antibody, and Buffers

G-17 and CA724 standard antigen and their paired antibodies (coating and detection antibodies) were obtained from Yidenuo Bio-technology (Guangzhou, China). Eu^3+^ and Sm^3+^ labeling reagents were purchased from PerkinElmer (Norwalk, USA). Washing buffer was as follows: 20 mmol/L Tris-HCl, 0.9% NaCl, and 0.05% Tween-20 (v/v), pH 8.0. Blocking buffer was as follows: 50 mmol/L PBS, 5% BSA (m/v), and pH 7.4. Labeling buffer was as follows: 50 mmol/L Na_2_HCO_3_-Na_2_CO_3_, 0.9% NaCl, and pH 9.0. Assay buffer was as follows: 50 mM Tris-HCl, 0.02% BSA, 0.05% Tween-20, 0.02% Proclin300, and pH 7.8. Enhancement solution was as follows: 0.1 mol/L acetate-phthalate, 0.1% Triton X-100, 20 *μ*mol/L *β*-naphthoyltrifluoroacetate (Sigma-Aldrich, USA), 50 *μ*mol/L tri-n-octylphosphine oxide (Sigma-Aldrich, USA), 0.5% glacial acetic acid, and pH 3.2. The above buffers were all prepared by ourselves.

### 2.2. Clinical Samples

The subjects performed the gastroscopy and biopsies of the gastric antrum and gastric body mucosa. Subjects who did not show histological signs of glandular atrophy and abnormal tissue changes at any site of the stomach were considered to be the healthy control samples (M/F 35/34; range of age 25-61 years). Subjects with only histological signs of glandular atrophy at any site of the stomach were considered to be atrophic gastritis samples (M/F 42/36; range of age 35-66 years). Subjects with abnormal tissue changes in the stomach and confirmed by pathological biopsy were considered to be patients with gastric cancer (I and II grade) (M/F 36/41; age range 38-69 years). The Institutional Review Board of Guangzhou Youdi Bio-technology Co., Ltd. approved this study, and all subjects gave written informed consent.

### 2.3. Coating Procedure

The anti-G-17 and anti-CA724 coating antibodies were prepared at concentrations of 2 *μ*g/mL. 100 *μ*L anti-G-17 and anti-CA724 coating antibodies were, respectively, added to 96-well microplate and incubated at 37°C for 2 h. After washing one time, the microplate was blocked with blocking buffer overnight at 4°C. Then, washed the microplate one time and dried in a vacuum, and then stored at 4°C.

### 2.4. Eu^3+^ and Sm^3+^ Labeling Procedure

Eu^3+^ and Sm^3+^ labeling procedure was performed according to the manufacturer's instructions. 1 mg G-17 detection antibodies were washed two times and suspended in 250 *μ*L of labeling buffer, and then 500 *μ*g Eu^3+^ chelates were added and incubated overnight at 4°C. Then, a Sephadex G50 column purified the Eu^3+^-labeled antibodies. After purification, the labeled antibodies were stored in 50 mM Tris-HCl buffer at 4°C. Similarly, CA724 detection antibodies were labeled with Sm^3+^.

### 2.5. Assay Procedure

Through optimizing the standards/sample volume, coating antibody volume/ratio, Eu^3+^/Sm^3+^-labeled antibody volume/ratio, reaction time, washing time, and enhancement solution volume, a one-step assay procedure was established. All the assay procedure was set in advance and preformed the automatic detection by the time-resolved analyzer (Auto DELFIA 1235, PerkinElmer). Briefly, 50 *μ*L serum samples or standards, 80 *μ*L Eu^3+^-labeled antibodies, and 80 *μ*L Sm^3+^-labeled antibodies were added into 96-wells plate and then incubated at room temperature for 40 min. After washing the wells 5 times, 200 *μ*L enhancement solution was added to the wells and shaken gently for 2 min. Finally, the time-resolved analyzer measured the fluorescence.

### 2.6. Standard Curves and Sensitivity Assay

The standards of G-17 and CA724 were diluted into (0, 0.1, 1, 10, 100, 500, and 1000 pg/mL) and (0, 0.1, 1, 10, 100, 500, and 1000 U/mL), respectively, and then were detected according to the optimized assay procedure. The log function values of G-17/CA724 standards concentrations were plotted as *X* axis, and the log function values of their relative light unit (RLU) as the *Y* axis performed a linear fit and draw a standard curve. 0 pg/mL and 0 U/mL dilutions were detected for 10 times and then calculated the mean values and standard deviation (SD): the sensitivity = mean + 2^∗^SD [18].

### 2.7. Specificity Assay

Some common serum interferents were selected for specificity assay, including serum albumin (SA), carcinoembryonic antigen (CEA), and carbohydrate antigen199 (CA199), interleukin 6 (IL-6), and tumor necrosis factor-*α* (TNF-*α*). High concentration interferents were added into the health control serum and detected using this TRFIA kit. The levels of these interferents in health control serum (basal concentration) were also detected using this TRFIA kit: crossreactivity (%) = (determined concentration − basal concentration)/interferents concentrations × 100.

### 2.8. Precision and Stability Assay

Firstly, three batches of TRFIA kits were produced for accuracy and stability assay. Then, three concentration levels (high, medium, low) of standard dilutions were added into the health control serum and detected their concentrations using the TRFIA kits and calculated the mean values and their SDs through six independent experiments: recovery (%) = (determined concentration − basal concentration)/spiked concentration × 100.CV (%) = SD/mean × 100.

### 2.9. Sensitivity and Accuracy Comparison with Commercial Kits

To compare this TRFIA method with the commercial G-17 chemiluminescence kit (registration certificate for medical device: Lu-20192400039, China) and registered CA724 electrochemiluminescence kit (Roche, registration certificate for medical device: 20183402635, Germany), parallel tests were performed simultaneously using the serum of the 69 health normal subjects, 78 subjects with atrophic gastritis, and 77 subjects with I/II grade gastric cancer. All detection steps were performed according to the manufacturer's guidance. The concentrations values of G-17/CA724 detected by this TRFIA were plotted as *X* axis, and the concentrations values of G-17/CA724 detected by the commercial registered kits were plotted as *Y* axis, which obtained the Pearson correlation coefficient (*r*).

### 2.10. Reference Interval

This TRFIA was used to detect the G-17 and CA724 concentrations of 69 health normal subjects, 78 subjects with atrophic gastritis, and 77 subjects with I/II grade gastric cancer, respectively, and calculated their G-17 and CA724 concentrations according to the standard curves. The concentration values performed a normality test with SPSS 17.0, respectively: cutoff = mean ± 1.96SD (bilateral), cutoff = mean − 1.64SD (unilateral lower limit), or cutoff = mean ± 1.64SD (unilateral upper limit) [19].

### 2.11. Statistical Analysis

Data were statistically analyzed and graphed using GraphPad Prism 5 (GraphPad Software, USA). All results are presented as the mean ± standard deviation (SD).

## 3. Results

### 3.1. Standard Curves and Sensitivity of the TRFIA Kit

The standard curves of G-17 and CA724 are presented in Figure 1. The standard curve equations were as follows: log*Y* = 0.583log*X* + 3.9239 (*R*^2^ = 0.9921) for G-17 and log*Y* = 0.5327log*X* + 3.6016 (*R*^2^ = 0.9915). The standard curves exhibited well-defined linear relationships between the wide-range analyze concentrations (0.1-1000) and fluorescence values. The sensitivity for G-17 was 0.54 pg/mL and for CA724 was 0.28 U/mL.

### 3.2. Specificity of the TRFIA Kit

This TRFIA kit detected the high concentrations of five interferents (SA, CEA, CA199, IL-6, and TNF-*α*) that was added into the health control serum, and the results are presented in Table 1. There was very low crossreactivity (all lower than 1%), indicating this TRFIA kit had high specificity and affinity for G-17 and CA724, and the common interferents could not affect the detection accuracy of this TRFIA kit.

### 3.3. Precision and Stability of the TRFIA Kit

The accuracy and stability of the TRFIA were assessed by detection the health control serum that had been spiked with G-17 (10, 100, and 500 pg/mL) and CA724 (1, 100, and 500 U/mL) standards. As is shown in Table 2, the average recoveries ranged from 100.52% to 110.30% for G-17 and 103.02% to 116.00% for CA724. All CVs of the intra- and interassay were below 10%. Table 2 results indicated that the accuracy and stability of this TRFIA were high and meet the requirements of clinical immunoassays.

### 3.4. Comparison Results of the TRFIA Kit

The concentrations of G-17/CA724 in 69 health normal subjects, 78 subjects with atrophic gastritis, and 77 subjects with I/II grade gastric cancer were statistically analyzed and graphed using GraphPad Prism 5. The comparison results are shown in Figure 2, and the Pearson *r* was 0.9117 for G-17 and 0.9449 for CA724. The high Pearson coefficient showed that this TRFIA method has a comparable detection performance to commercial kits.

### 3.5. Reference Intervals of the TRFIA Kit

The concentrations values of G-17 and CA724 in three different populations are in accordance with the normality distribution, and the cutoff values are shown in Table 3. For the health subjects, the cutoff value of G-17 was 88.41 pg/mL and 5.47 U/mL for CA724. For the subjects with atrophic gastritis, the cutoff value of G-17 ranged from 67.89 to 334.30 pg/mL and 0.65 to 5.75 U/mL for CA724. For the subjects with I/II grade gastric cancer, the cutoff value of G-17 was 138.65 pg/mL and 8.01 U/mL for CA724.

## 4. Discussion

Gastric carcinoma (GC) is one of the most common malignancies in the world, and it keeps a high incidence in many countries, such as China [20]. Owing to its poor outcome, GC presents one of the great early screening and therapeutic challenges [21]. Atrophic gastritis is the main precursor lesions of gastric cancer. Dynamic monitoring of atrophic gastritis and early gastric cancer markers is necessary to predict the development of the gastric diseases. The previous studies indicate that none of the tumor markers was organ-specific [22]. The addition of any one tumor marker assay consistently improved the diagnostic accuracy. Clinical sample research found that G-17 and PG can be potent markers in screen of diagnosis of early gastric cancer, and G-17 combined with PG can improve the sensitivity and accuracy to 96.2% [23]. Sensitivity of serum CA724 is limited, and combination detection (e.g., CA724 + CEA + CA199) is considerable to improve sensitivity without impairing specificity [11]. Therefore, we selected G-17 and CA724 as the markers and established a new combination detection method to predict the development of the gastric diseases.

The existing detection methods for G-17 and CA724 include ELISA, immunochromatography, immunoturbidimetry, and chemiluminescence [24]. The high-sensitivity immunoassay of early tumor markers plays an important role in early screening and disease monitoring and are attracting more and more attention [24, 25]. Among varieties of immunoassays, TRFIA is a new detection method with a wide detection range and high sensitivity. TRFIA employs the lanthanide chelate europium (Eu^3+^) and samarium (III)- (Sm^3+^-) labeled paired antibodies which possess a high fluorescence intensity and virtually no background resulting in a highly sensitive detection method [26]. The resultant wider assay dynamics enabled us to analyze a large panel of serum samples [27]. In this study, we established a highly sensitive and wide range TRFIA method to detect G-17 and CA724 simultaneously in serum, and this TRFIA can be used for predicting the development of the gastric diseases.

The application of the immunoassay in further depends on three important parameters including specificity, repeatability, and stability. For this TRFIA method, it has low crossreactivity (all lower than 1%) with five interferents (SA, CEA, CA199, IL-6, and TNF-*α*). The average recoveries ranged from 100.52% to 110.30% for G-17 and 103.02% to 116.00% for CA724. All CVs of the intra- and interassay were below 10%. The above three parameters met the requirements specified of the clinical in vitro diagnostic reagents. Furthermore, Pearson correlation analysis was carried out to evaluate the difference between our TRFIA method and the commercial kits, and the Pearson *r* was 0.9117 for G-17 and 0.9449 for CA724 indicating that this TRFIA method has a comparable detection performance to commercial kits.

The diagnostic accuracy is primarily affected by the validity of the reference interval of the related indicators [28]. Each detection method must establish its own reference interval. As far as we know, no studies have validated the reference value of G-17 and CA724 used to discriminate health, atrophic gastritis, and early gastric cancer. In this study, through the detection of G-17 and CA724 in 69 health normal subjects, 78 subjects with atrophic gastritis, and 77 subjects with I/II grade gastric cancer, we obtained the reference intervals of G-17 and CA724 for this TRFIA method: when G − 17 < 88.41 pg/mL and CA724 < 5.47 U/mL, the subject is healthy and has a low risk of gastric cancer; when G − 17 ≥ 138.65 pg/mL and CA724 ≥ 8.01 U/mL, the subject has the possibility of transforming from atrophic gastritis to early gastric cancer.; when G-17 was 67.89 to 334.30 pg/mL and CA724 was 0.65 to 5.75 U/mL, the subject may simply have atrophic gastritis. However, due to the small sample size, these reference intervals are not completely accurate and reliable. Therefore, to confirm the precise values of these optimal cutoff values, larger population-based cohort studies should be conducted.

In conclusion, we established a TRFIA method to detect the concentrations of G-17 and CA724 in serum. The TRFIA has high accuracy and precision and was comparable with commercial kits in the determining of clinical serum samples, indicating that the determining performance of this TRFIA method met the requirements specified of the clinical in vitro diagnostic reagents. In short words, this TRFIA provides a new method for sensitive, accurate, and specific early screening of gastric cancer.

## Figures and Tables

**Figure 1:** The standard curves of G-17 and CA724. The log function values of G-17/CA724 standards were plotted as *X* axis, and the log function values of their relative light unit (RLU) as the *Y* axis performed a linear fit and draw the standard curves.

**Figure 2:** Correlation of G-17 and CA724 levels between this TRFIA and the commercial kits. The concentration values of G-17 or CA724 detected by this TRFIA were plotted as *X* axis, and the concentration values of G-17 or CA724 detected by the commercial kits were plotted as *Y* axis, which performed a Pearson correlation analysis and obtained the Pearson correlation coefficient (*r*).

**Table 1:** Specificity results of the TRFIA kit.

Interferents (500 ng/mL)	Determined indicator	Determined concentrations	Basal concentration	Crossreactivity (%)
SA	G-17	52.60 ± 2.82	48.22 ± 2.71	0.876
	CA724	4.94 ± 0.42	3.76 ± 0.45	0.236
CEA	G-17	49.63 ± 2.24	48.22 ± 2.71	0.282
	CA724	5.12 ± 0.46	3.76 ± 0.45	0.272
CA199	G-17	53.12 ± 2.34	48.22 ± 2.71	0.98
	CA724	4.85 ± 0.40	3.76 ± 0.45	0.218
IL-6	G-17	52.34 ± 2.40	48.22 ± 2.71	0.824
	CA724	4.08 ± 0.41	3.76 ± 0.45	0.064
TNF-*α*	G-17	51.31 ± 2.69	48.22 ± 2.71	0.618
	CA724	4.99 ± 0.38	3.76 ± 0.45	0.246

**Table 2:** Accuracy and recovery of this TRFIA.

Indicators	Spiked concentration	Intra-array (*n* = 6)			Interarray (*n* = 6)		
		mean ± SD	Recovery (%)	CV (%)	mean ± SD	Recovery (%)	CV (%)
G-17 (pg/mL)	10	59.25 ± 3.51	110.30	5.92	59.27 ± 3.96	110.50	6.68
	100	156.34 ± 8.25	108.12	5.27	154.69 ± 9.24	106.47	5.97
	500	564.31 ± 13.22	103.22	2.34	570.16 ± 15.28	104.39	2.68

CA724 (U/mL)	1	4.82 ± 0.41	106.00	8.51	4.92 ± 0.48	116.00	9.76
	100	106.35 ± 5.61	102.59	5.27	108.68 ± 7.41	104.92	6.82
	500	506.37 ± 18.38	100.52	3.63	518.84 ± 20.27	103.02	3.91

**Table 3:** The cutoff values of health normal subjects, subjects with atrophic gastritis, and subjects with I/II grade gastric cancer by this TRFIA.

Subjects	Indicators (ng/mL)	Mean	SD	Formula	Cutoff (pg/mL or U/mL)
Health normal	G-17	64.3	14.7	Mean + 1.64SD	88.41
	CA724	3.5	1.2		5.47

Atrophic gastritis	G-17	150.8	42.3	Mean ± 1.96SD	67.89~334.30
	CA724	3.2	1.3		0.65~5.75

I/II grade gastric cancer	G-17	233.21	57.66	Mean − 1.64SD	138.65
	CA724	12.93	3.00		8.01

## Data Availability

The datasets used and/or analyzed during the current study appear in the submitted article.
